The article "Comparison of Curative Complications between Mammotome-Assisted Minimally Invasive Resection and Conventional Open Resection for Breast Neoplasm: A Retrospective Clinical Study" was retracted in 2024. Reasons: signs of a paper mill; suspected computer-generated content; unreliable results or conclusions; concerns about the data.

# Comparison of Curative Complications between Mammotome-Assisted Minimally Invasive Resection and Conventional Open Resection for Breast Neoplasm: A Retrospective Clinical Study

**DOI:** 10.1155/2021/7739628

**Published:** 2021-11-17

**Authors:** Rui Li, Jingyan Li, Shanzheng Chen, Binglan Xiao, Lihua Liu, Ning Zhu

**Affiliations:** ^1^Loudi City Central Hospital, Loudi, 417000 Hunan, China; ^2^Hunan University of Medicine, Huaihua, 418000 Hunan, China

## Abstract

**Background:**

To know the clinical value of mammotome-assisted minimally invasive resection (MAMIR) in the treatment of patients with breast neoplasm, we performed a retrospective clinical study for the patients treated with the MAMIR and conventional open resection (COR).

**Methods:**

Postoperative complications were compared between 40 patients treated with the MAMIR and 40 patients treated with the COR. The postoperative complications mainly included intraoperative blood loss, hospitalization days, operative time, surgical scar, and incidence of postoperative complications.

**Results:**

We found that the amount of intraoperative blood loss, hospitalization days, operative time, surgical scar, and incidence of postoperative complications in the MAMIR group were significantly lower than those of patients in the COR group.

**Conclusion:**

Our results indicated that patients with breast neoplasm treated with the MAMIR had better outcomes, which reinforced the advantage of this approach.

## 1. Introduction

Breast neoplasms are a wide spectrum of pathologies from benign proliferations, high-risk lesions, precursor lesions, to invasive malignancies. Breast cancer is the most commonly diagnosed cancer and the leading cause of cancer death [1]. In 2020, there were almost 2.3 million new breast cancer cases and 0.68 million breast cancer deaths [1]. Surgery is a common treatment for cancers, including breast cancers [2–4]. Most patients with breast cancer who undergo surgery also need additional treatments, such as chemotherapy, hormone therapy, or radiation [5–7]. Breast cancer is the most common type of cancer with high incidence [1]. However, most breast neoplasm patients are determined to be noncancerous [8]. Breast neoplasm is a relatively common disease in women, which is more common in women of reproductive age, including benign tumors and malignant tumors. Although those benign tumors do not invade the surrounding tissue, they will interfere with the function of the breast if they are not surgically removed. Therefore, no matter if the patient's breast tumor is benign or malignant, surgical resection is necessary [9, 10]. Mammotome minimally invasive mastectomy is a minimally invasive mastectomy for breast masses under the guidance of ultrasound and according to the relevant principle of vacuum negative pressure suction [11–13]. It has the advantages of high accuracy of positioning, less bleeding, and better aesthetic appearance [13–15]. To know the clinical value of the mammotome-assisted minimally invasive resection (MAMIR) in the treatment of patients with breast neoplasm, we performed a retrospective comparative analysis of MAMIR and conventional open resection (COR) in the present study.

The article "Comparison of Curative Complications between Mammotome-Assisted Minimally Invasive Resection and Conventional Open Resection for Breast Neoplasm: A Retrospective Clinical Study" was retracted in 2024. Reasons: signs of a paper mill; suspected computer-generated content; unreliable results or conclusions; concerns about the data.

## 2. Materials and Methods

### 2.1. Object

This study was approved by the Ethics and Research Committees of Loudi City Central Hospital (Loudi, China) and was conducted in accordance with the principles outlined in the Declaration of Helsinki. We collected 80 patients who underwent breast resection treatment in our department from May 2019 to May 2021 for this retrospective study, of which there were 40 patients treated with MAMIR and 40 patients treated with COR.

*Measurement of breast tumor size*: Siemens Acuson S3000 Ultrasound Machine was used to diagnose the tumor size before the surgery, and the transverse and longitudinal diameters of tumors were measured in millimeters. *Measurement of surgical incision size*: at the first dressing change after surgery, a millimeter ruler was used to measure surgical incision size (accurate to millimeter).

### 2.2. Inclusion/Exclusion Criteria

*Inclusion criteria*: (1) patients should be diagnosed as benign or potentially benign by physical examination, color ultrasound, mammography, and histopathology according to bi-RADS classification criteria; (2) the maximum diameter of the patient's tumor should be less than 30 mm; and (3) both the patient and the patient's family members need to have read and signed the informed consent, which was reviewed and confirmed by the medical ethics committee.

*Exclusion criteria*: (1) patients whose preoperative pathological properties are not clear or suspected to be breast cancer or whose postoperative pathological diagnosis is malignant tumor; (2) patients with breast implants; (3) patients with contraindications to surgery; (4) the patient's maximum tumor diameter was greater than 30 mm; and (5) patients with hemangioma, coagulopathy, mental disorders, and other diseases need to be excluded.

### 2.3. Operative Method

*Conventional open resection*: after anesthesia is administered, the nipple is treated as the center to form a radial or arcuate surgical incision around the areola. The incision length is 2-4 cm. The skin, fat, and glands were incised and separated around the neoplasm to expose the neoplasm. The mass and surrounding normal tissue were excised, sutured, and bandaged.

The article "Comparison of Curative Complications between Mammotome-Assisted Minimally Invasive Resection and Conventional Open Resection for Breast Neoplasm: A Retrospective Clinical Study" was retracted in 2024. Reasons: signs of a paper mill; suspected computer-generated content; unreliable results or conclusions; concerns about the data.

*Mammotome-assisted minimally invasive resection*: according to the location of the patient's neoplasm, the appropriate posture was selected, the patient's back was properly padded, local anesthesia was carried out, and the surgical site was exposed. The needle insertion direction was determined according to the ultrasonic examination results. The incision length was 4 mm, hidden in the areola, midaxillary line, and lower margin of the mammary gland. Guided by B-ultrasound, a rotating breast cutter was placed below the lesion. The grooves of the rotary knife are aligned with the lesion, and the lesion is rotated and the specimen is extracted. After the tumor was completely resected with B-ultrasound, pressure hemostasis was performed. After 10-20 minutes of pressure, we cover with a bandage. The elastic bandage was applied with pressure for 48-72 hours.

### 2.4. Statistical Analysis

IBM SPSS 22 software is used for statistical analysis. A chi-square test is used for counting data, and *t*-test is used for measurement data. Data were presented in the form of mean ± SEM.

## 3. Results

### 3.1. Comparison of Clinical Features

We collected 40 patients who underwent MAMIR and 40 patients who underwent COR in our department from May 2019 to May 2021. There was no significant difference in age between the MAMIR group and the COR group (Figure 1(a)). However, the tumor size of patients treated with MAMIR was significantly smaller than that of patients treated with COR (Figure 1(b)).

### 3.2. Comparison of Clinical Complications

We performed the comparison analyses for the clinical complications, including the amount of intraoperative blood loss, hospitalization days, operative time, and surgical scar in the MAMIR group and the COR group. The results indicated that the amount of intraoperative blood loss in the MAMIR group was significantly reduced by about 50% (Figure 2(a)). Both the hospitalization days and the operative time of patients treated with MAMIR were significantly lower than those of patients treated with COR (Figures 2(b) and 2(c)). Spontaneously, we also found that the size of the surgical scar was also significantly smaller in the MAMIR group (Figure 2(d)).

We previously found that the tumor size in the MAMIR group was significantly smaller than that in the COR group. Then, we performed the correlation analyses for the amount of intraoperative blood loss, hospitalization days, operative time, and surgical scar with the treatment manner. The results indicated that the treatment manner was correlated with the intraoperative blood loss, hospitalization days, operative time, and surgical scar (Figure 2(e)).

The article "Comparison of Curative Complications between Mammotome-Assisted Minimally Invasive Resection and Conventional Open Resection for Breast Neoplasm: A Retrospective Clinical Study" was retracted in 2024. Reasons: signs of a paper mill; suspected computer-generated content; unreliable results or conclusions; concerns about the data.

### 3.3. Comparison of Postoperative Complications

Additionally, we also performed the comparison analyses for the postoperative complications, including local hematoma, fat liquefaction, and infection. In the COR group, we found 2 cases of local hematoma, 3 cases of fat liquefaction, and 1 case of infection. In the MAMIR group, we found 1 case of local hematoma. The chi-square test showed no significant difference between them (Table 1).

Subsequently, we performed the chi-square for all postoperative complications, and found that the total rate of postoperative complications in the MAMIR group was 2.5%, which was significantly lower that of the COR group (15%) (Table 2).

## 4. Discussions

Breast neoplasm is a relatively common disease in women. Surgical resection of breast masses is often performed clinically. However, it is difficult to remove a small breast mass with traditional open surgery. In addition, the incision is relatively large, leaving a large scar on the breast, which is not easy to be accepted by patients with breast tumors [16, 17]. Mammotome minimally invasive mastectomy is a minimally invasive mastectomy for breast masses under the guidance of ultrasound and according to the relevant principle of vacuum negative pressure suction [11–13]. It has the advantages of high accuracy of positioning, less bleeding, and better aesthetic appearance [13–15].

To know the clinical value of MAMIR and COR for the treatment of patients with breast neoplasm, we performed comparison analyses for 40 patients who underwent mammotome minimally invasive surgery and 40 patients who underwent conventional open surgery. We found that the amount of intraoperative blood loss, hospitalization days, operation time, and surgical scar in the test group were significantly lower than those in the control group. The total rate of postoperative complications in the mammotome minimally invasive surgery group was significantly better than that of the conventional open surgery group. Our results suggest that minimally invasive mastectomy is better in treating breast tumors than traditional open surgery, which reinforced the advantage of the surgery treatment [18–20].

## Figures and Tables

**Figure 1:** Comparison of clinical features. (a) Comparison of age in patients treated with the MAMIR and COR. (b) Comparison of tumor size in patients treated with the MAMIR and COR. MAMIR, *n* = 40; COR, *n* = 40. ^∗^*p* < 0.05, ^∗∗^*p* < 0.01, ^∗∗∗^*p* < 0.001.

**Figure 2:** Comparison of clinical complications. (a–d) Comparison of intraoperative blood loss (a), hospitalization days (b), operative time (c), and surgical scar (d) in patients treated with the MAMIR and COR. (e) Correlation analyses of treatment manner with the clinical complications. MAMIR, *n* = 40; COR, *n* = 40. ^∗^*p* < 0.05, ^∗∗^*p* < 0.01, ^∗∗∗^*p* < 0.001.

The article "Comparison of Curative Complications between Mammotome-Assisted Minimally Invasive Resection and Conventional Open Resection for Breast Neoplasm: A Retrospective Clinical Study" was retracted in 2024. Reasons: signs of a paper mill; suspected computer-generated content; unreliable results or conclusions; concerns about the data.

**Table 1:** Local hematoma/fat liquefaction/infection comparison.

Group	Local hematoma		Fat liquefaction		Infection comparison	
	No	Yes	No	Yes	No	Yes
COR	38	2	37	3	39	1
MAMIR	39	1	40	0	40	0
*X* ^2^	0.346		3.117		1.013	
*p*	0.556		0.077		0.314	

**Table 2:** Postoperative complication comparison.

Group	Local hematoma & fat liquefaction & infection comparison	
	No	Yes
COR	34	6
MAMIR	39	1
*X* ^2^	3.914	
*p*	0.048	

## Data Availability

The datasets generated and analyzed for the current study are available.
